# Emergency Endovascular Interventions on Descending Thoracic Aorta: A Single-Center Experience

**DOI:** 10.1155/2023/6600035

**Published:** 2023-01-03

**Authors:** Piotr Buczkowski, Mateusz Puslecki, Marcin Ligowski, Marek Dabrowski, Sebastian Stefaniak, Zuzanna Fryska, Jerzy Kulesza, Robert Juszkat, Marek Jemielity, Bartlomiej Perek

**Affiliations:** ^1^Department of Cardiac Surgery and Transplantology, Cardiac and Thoracic Surgery, Poznan University of Medical Sciences, Dluga Street 1/2, Poznan 61–848, Poland; ^2^Department of Medical Rescue, Emergency Medicine, Poznan University of Medical Sciences, Collegium Adama Wrzoska, Rokietnicka Street 7, Poznan 60-806, Poland; ^3^Polish Society of Medical Simulation, Slupca, Poland; ^4^Department of Medical Education, Poznan University of Medical Sciences, Collegium Adama Wrzoska, Rokietnicka Street 7, Poznan 60-806, Poland; ^5^Faculty of Medicine, Poznan University of Medical Sciences, Poland; ^6^Department of Radiology, Poznan University of Medical Sciences, Dluga Street 1/2, Poznan 61–848, Poland

## Abstract

**Background:**

Implementation of emergency endovascular aortic repair provides an attractive opportunity in the treatment of complicated acute aortic syndromes involving descending aorta.

**Aim:**

The aim of this study was to analyze the effectiveness of thoracic endovascular aortic repair (TEVAR) for the treatment of acute surgical emergencies involving the descending thoracic aorta.

**Methods:**

A retrospective review of the medical records of all patients undergoing TEVAR in a single center since 2007 was undertaken. Patients with the aortic disease treated on emergency inclusion criteria were complicated spontaneous acute aortic syndrome (csAAS), traumatic aortic acute injuries (TAIs), and other indications requiring emergent intervention. Technical and clinical success with patient mortality, survival, and reoperation rate was evaluated according to Society for Vascular Surgery reporting standards for thoracic endovascular aortic repair (TEVAR).

**Results:**

The emergency interventions were necessary in 74 cases (51.0%), including patients with the complicated spontaneous acute aortic syndrome (csAAS) (64.8%; *n* = 48) and traumatic aortic acute injuries (TAIs) (31.1%). In addition, in one case aortic iatrogenic dissection (AID) and in 2 other fistulas after the previous stent graft, implantations were diagnosed. All procedures were done through surgically exposed femoral arteries while 2 hybrid procedures required additional approaches. The primary technical success rate was 95.9%, in 3 cases endoleak was reported. The primary clinical success occurred in 94.5%. All patients survived the endovascular interventions, whereas during in-hospital stay one of them died due to multiorgan failure (early mortality 1.3%). During the follow-up period, lasting 6 through 164 months (median 67), 11 patients died. Annual, five- and ten-year probability of survival was 86.4 ± 0.04%, 80.0 ± 0.05%, and 76.6 ± 0.06%, respectively. However, the rate of 5-year survivors was significantly higher after TAI (95.2%) than scAAS (63.4%) (*p*=0.008). Early after the procedure, one individual developed transient paraparesis (1.3%). No other serious stent-graft-related adverse events were noted within the postdischarge follow-up period.

**Conclusions:**

Descending aortic pathologies requiring emergent interventions can be treated by endovascular techniques with optimal results and low morbidity and mortality in an experienced and dedicated team.

## 1. Introduction

Thoracic endovascular aortic repair (TEVAR) initially developed for elective procedures has also become an attractive method of treating acute descending aortic syndromes (AASs) in emergency indications. Conventional open surgery is associated with high perioperative mortality and morbidity. TEVAR application led to a positive decline in the operative mortality and morbidity. The most common forms with poor prognosis and the necessity of emergent interventions are complicated aortic dissection and disruption [1, 2]. Complicated aortic type B dissections (cTBDs) are associated with a 25–50% mortality within 48 hours [1, 2]. The damage of the heart and large vessels, including traumatic aortic injuries (TAIs), consist of the second cause of multiorgan trauma-related deaths and is diagnosed in more than 30% of victims of serious blunt thoracic injuries. The consequences of complicated AAS such as hemorrhage, hypovolemic shock, or organ and tissue malperfusion make AAS as life-threatening conditions [3].

Acute aortic diseases, particularly those confining also descending part, must be considered as an interdisciplinary entity that should involve specialists in surgery (both cardiac and vascular), interventional radiology, anesthesiology, and cardiology. Such approach through the acceleration of the diagnostic and therapeutic process of critically ill patients with multiorgan trauma directly translates into the results of treatment and final outcomes.

This is the first single-center retrospective, observational, cohort study that provides technical and clinical success according to Society for Vascular Surgery reporting standards for thoracic endovascular aortic repair (TEVAR) [4]. Moreover, the safety criteria of the TEVAR procedure adopted strictly in our center and meeting the recommendations of the Tokyo Consensus including minimal proximal and distal Landing Zone—20 mm (since 2019–25 mm) may be responsible for the high rate of technical and clinical success [5, 6].

The aim of this study was to analyze the effectiveness of thoracic endovascular aortic repair (TEVAR) for the treatment of acute surgical emergencies involving the descending thoracic aorta catastrophes.

## 2. Methods

### 2.1. Study Design

A retrospective review of the medical records of all patients undergoing TEVAR in a single center since 2007 was undertaken Since 2007, 145 patients with descending aorta pathologies have been treated by TEVAR in the Department of Cardiac Surgery and Transplantology, a center that served as referential TEVAR center for nearly 5 million of inhabitants. Among them, in 74 cases (51%), the emergency TEVAR procedures, defined as emergent interventions (starting before the beginning of the next working day) were performed. Patients with the aortic disease treated on an emergency inclusion criteria were complicated spontaneous acute aortic syndrome (csAAS), traumatic aortic acute injuries (TAIs), and other indications requiring emergent intervention. Patients with elective descending aorta aneurysm (DAA), uncomplicated Type B aortic dissections, and requiring elective TEVAR reinterventions were excluded. The STROBE checklist (Figure 1) is applied in this study.

According to the rules of the Local Bioethical Committee of our university, the Statement of Ethics Approval is not required for retrospective data analysis of patients treated with the use of the standard and accepted methods.

### 2.2. Main Variables of Interest

From each patient we collected preoperative information, specific data according to the indication of repair, intraoperative data, and postoperative data. Technical and clinical success with patient mortality, survival, and reoperation rate were evaluated according to Society for Vascular Surgery reporting standards for thoracic endovascular aortic repair (TEVAR) [4]. We specifically analyzed the emergency indication for each disease condition: complicated spontaneous acute aortic syndrome (csAAS), traumatic aortic acute injuries (TAIs), and other indications requiring emergent intervention.

These clinical complications were: infection, postoperative bleeding requiring repeat surgery, postoperative paraplegia, cerebrovascular accident (CVA), acute coronary events, renal failure with a need for dialysis, respiratory failure, and intestinal ischemia. We also analyzed survival at 30 days and 6–164 months follow-up period.

### 2.3. Postoperative Evaluation

The approval in the Department protocol after thoracic stent graft implantation included physical examinations completed by computed tomographic angiography (CTA) at 1, 3, 6, and 12 months after the procedure and later on once a year. Patients who had the hybrid procedures were additionally followed up every 3 months for the first 3 years.

### 2.4. Definitions

- *Emergent Interventions.* Operation before the beginning of the next working day after the decision to operate (EuroSCORE).
- *Critical Preoperative State*. ≥1 of the following in the same hospital admission as the operation: ventricular tachycardia or fibrillation or aborted sudden death; cardiac massage; ventilation before arrival to OR; inotropes; IABP or VAD before arrival to OR; acute renal failure, defined as anuria or oliguria <10 mL/hr (EuroSCORE).
- *Post-Implantation Syndrome (PIS).* The Velazquez syndrome, called also postimplantation syndrome (PIS), was defined by the presence of leukocytosis (>12,000 leukocytes/*μ*L) and the occurrence of fever (>38°C–auricular temperature) but without following markers of infection such as increased concentrations of high sensitivity C-reactive protein and procalcitonin when infectious complications were excluded (no clinical evidence of infection, negative blood cultures, and absence of local complications of the surgical wound) [4].
- *Primary Technical Success.* This is defined on an intent-to-treat basis that begins with the implantation procedure and requires the successful introduction and deployment of the device in the absence of surgical conversion to open repair, death <24 hours, type I or III endoleaks as evidenced by procedural angiography, or graft obstruction [4].
- *Primary Clinical Success.* This can only occur without any of the following: death as a result of treatment or as a result of the original pathology that was treated; type I or III endoleak, infection, or aortic thrombosis; aneurysm expansion (diameter >5 mm, volume >10% or greater than two times interobserver variability) or rupture; conversion to open repair; or failure to arrest the original pathologic process (e.g., embolization from penetrating ulcer) or causing a new thoracic aortic pathology as a result of the intervention (e.g., pseudoaneurysm, dissection, and intramural hematoma) [4];
- *Secondary Clinical Success*: This is defined as clinical success obtained initially but temporarily interrupted by a failure that is corrected with the use of an additional, secondary surgical procedure; for example, a type I endoleak develops in an initially excluded aneurysm due to endograft migration at 2 years and is corrected by placement of a new, more proximal endograft. Conversely, clinical failure includes death as a result of treatment or as a result of the original pathology that was treated or a pathology caused by the initial procedure (e.g., aneurysm rupture, or dissection extending to cause mesenteric ischemia and resulting in death), type I or III endoleak, graft migration, infection, or thrombosis, aneurysm expansion (as defined elsewhere in this document; aneurysm rupture), conversion to open repair, failure to arrest the original pathologic process, or appearance of a new thoracic aortic pathology as a result of intervention [4];

### 2.5. Principal Procedure: Stent-Graft Implantation

All endovascular procedures were performed by the experienced team of two cardiac surgeons and one interventional radiologist, mostly in the vascular intervention room. An exception was two complex procedures carried out in the hybrid room with the assistance of a vascular surgeon. In addition, all but two were treated under general anesthesia. These two patients had to undergo procedures with local anesthesia and sedation but without endotracheal intubation because of diagnosed tracheal injury. Standard antibiotic prophylaxis was used and all patients obligatory received 5,000 IU of heparin. An exception was one patient after trauma with a fracture of the skull base. In all cases, a stent graft was implanted by means of a femoral surgical approach through the right common femoral artery. The left femoral artery was punctured percutaneously by Seldinger's technique for the introduction of a 6F straight catheter with side holes on a pigtail 5F one in the ascending aorta to position the landing zone target. The stent grafts were placed in the thoracic aorta over an Amplatz 0.35 guidewire. DSA (Digital Subtraction Angiography) was performed in five to ten series with the use of an ionic contrast medium to confirm the final position and tightness of the prosthesis.

### 2.6. Adjunctive Procedure: Hemi-Arch Transposition

In two cases, after CT examination analysis multidisciplinary team decided to perform a two-step procedure in a hybrid room. After carotid-to-carotid anastomoses with FEP Ringed GORE-TEX STRETCH (Gore & Associates, Flagstaff, Arizona, USA) vascular graft prostheses (8 mm in diameter), eventually the stent grafts were implanted distally to brachiocephalic trunk but covering the orifices of both the left common carotid and left subclavian arteries.

### 2.7. Statistical Analysis

The quantitative variables were checked for normality distribution with the use of the Shapiro–Wilk W test. If they met normal distribution they were presented as mean with standard deviation, otherwise as median with range (minimum; maximum). Categorical variables were expressed as the numbers (*n*) with percentages (%). The probability of survival was stratified according to the Kaplan–Meier method and if applicable, compared by means of the Cox F test. *p* value less than 0.05 was considered to indicate differences of statistical significance. The statistical analysis was performed by the use of Statistica 13.3 (TIBCO Software Inc., 2017, USA).

## 3. Results

### 3.1. Patients

This study involved 74 patients with emergent TEVAR including 48 (64.8%) patients with complicated spontaneous AAS (csAAS), including complicated typical TBD (cTBD) (*n* = 23; 31.1%), the same number with ruptured descending thoracic aortic aneurysms (RTAA) and 2 (2.7%), one with penetrating atherosclerotic ulcers (PAU) and one intramural hematoma (IH). In 23 cases (31.1%) indication for emergent TEVAR was (31.1%) TAI, and among them 14 with traumatic aortic disruption (TAD). In one case aortic iatrogenic dissection (AID) with mesenteric ischemia and in the other 2 subjects aorto-oesophageal fistulas were the other indications for emergent TEVAR. The baseline characteristics of all patients are outlined in Table 1, whereas indications for emergency TEVAR together with some procedural details are in Table 2.

In the majority of patients, Zenith stent grafts (Cook Inc., USA) were implanted. In one case Jotec (JOTEC GmbH, Stuttgart, Germany) and in the other four GORE (Gore Medical, Flagstaff, USA) stent grafts were used (Zenith *n* = 69; GORE *n* = 4; JOTEC *n* = 1). The mean prostheses diameter was 33.1 ± 5.2 mm, whereas the length was 161.7 ± 27.1 mm, respectively. Single stent grafts were used in 70 cases; two stents in 4 patients. In 38 cases, the proximal graft landing zone was below the orifice of the left subclavian artery (LZ 3 and 4), in the other 34 (45.9%) the prosthesis covered the orifice of the left subclavian artery (LZ 2). In 2 subjects operated on in the hybrid room, the landing zone was more proximal (LZ 1) and it was forced to cover the left common carotid artery. Intraprocedural data with a 95.9% primary technical success rate are presented in detail in Table 2.

### 3.2. Intraoperative Results

All patients survived the endovascular interventions, whereas during in-hospital stay one of them died due to multiorgan failure (early mortality 1.3%). During in-hospital stays in 3 cases, endoleak type I was reported and the primary clinical success occurred in a final rate of 94.5% [4].

### 3.3. Initial 30-Day Clinical Success

One of the patients died during an in-hospital stay as a consequence of multiorgan failure (early mortality rate 1.3%) on the 19th postoperative day. The patient was operated on due to aorto-oesophageal fistulas but developed sepsis that eventually led to fatal MOF and death. The second patient after primary TEAR presented a severe stroke, never left the hospital, and died 46 days after the procedure. The TEVAR related deaths in total was 2.6% (Table 3).

Early after procedures, one patient developed transient paraparesis (*n* = 1, 1.3%), 2 individuals strokes (2.6%) and in 3 cases type I endoleaks were noted. The total prevalence of early neurological adverse events was 4.0%. In one case we observed hemodynamically nonsignificant endoleak and he was discharged in good clinical status and remained asymptomatic, and with a stable view in the follow-up CTA examinations, two next patients were qualified for reintervention. In 18 cases there was a necessity to put the drain to the left pleural cavity, but a few days after TEVAR. Notably, preprocedural bleedings were the predominant reasons. Fifty percent of patients experienced Velazquez postimplantation syndrome (PIS) in the early postprocedural period. No other complications associated with the implantation of the stent graft during the perioperative period were noticed. In our group, the median length of stay in the intensive care unit (ICU) was 1 day, whereas the total hospitalization time was 6 days.

### 3.4. Long-Term Clinical Success Follow-Up Results

During the postdischarge follow-up period that lasted 6 through 164 months (median time 67), 11 patients died. Annual, five- and ten-year probability of overall survival was 86.4 ± 0.04%, 80.0 ± 0.05%, and 76.6 ± 0.06%, respectively. However, the rate of 5-year survivors was significantly higher after TAI (95.2 ± 3.2%) than csAAS (63.4 ± 5.9%) (*p* = 0.001) (see Figures 2(a) and 2(b)).

Two of the patients needed further TEVAR reintervention, one in 14 months of observation and the second in 5 years after primary TEVAR. No other serious stent-graft-related adverse events, infection, or migration were noted during the follow-up period (Tables 3 and 4). The secondary clinical success rate was 93.2% (Table 3) [4].

## 4. Discussion

TEVAR initially developed for elective interventions in the treatment of the degenerative aneurysms quickly became also to be a technique of choice for emergency cases. Such a wide application of the techniques allowed to reduce the mortality associated with these diseases, as well as the associated risk of open surgery. Emergency lesions of the thoracic aorta, including csAAS, TAI, or complicated aorto-oesophageal fistulas are challenging. The emergency conventional repair of these conditions is associated with high morbidity-mortality, and despite the advances in surgical techniques and perioperative management, this type of surgery continues to pose a very high risk [7, 8]. Endovascular techniques have become the option of choice in emergency situations since the morbidity-mortality reported in the literature is favorable to these techniques versus classical [7, 8]. Recent meta-analyses of 14,580 patients confirmed better perioperative outcomes with TEVAR compared to the classical approach. However, there are still not many research data devoted to the assessment of 10-year survival and outcomes after endovascular procedures [7].

### 4.1. Emergency Indications for TEVAR and Outcomes

Our early results in TAI subgroup, mortality rate of 0% and a low risk of neurological complications are favorable and comparable or to the previous studies. For example, Richens et al. reported 7,768 patients who underwent TEVAR in TAD with early mortality of 9% and a neurological complications of 3% [9–11]. In contrast, open TAD surgery is associated with a mortality rate in excess of 28% with a neurological risk of close to 30%. In the case of the TAI in our series, 39.1% were of type III and 60.9% of type IV according to the Azizzadeh classification endorsed by the Society of Vascular Surgery (SVS) [4, 12]. European Society for Vascular Surgery (ESVS) recommends emergency repair in such situations (recommendation 27: class I, level of evidence C) [11, 13]. The final decision for urgent or delayed intervention repair should be based on the cumulative risk of aortic rupture and additional injuries. The minimal invasive endovascular TEVAR are attractive and beneficial for emergency treatment of unstable patients, received less blood transfusion, and manifested lower mortality rate and shorter in-hospital stay [6]. Up to now, there are scared data about long-term follow-up outcomes involving a period 10–15 years assessing function of implanted stent-graft in TAI. We did show in our analysis excellent primary and secondary clinical success and long-term outcomes, 95% probability of 10-year survival after TAI treated by means of emergent TEVAR, additionally in the most severe injuries (type III and IV). Our results are comparable with the highest volume TEVAR comparison with open surgery in TAI cases, reported by Demetriades and colleagues. The TEVAR group patients received less blood transfusion and manifested a lower mortality rate and shorter in-hospital stay (6). TAI is a specific traumatic disease of the previously healthy aorta that can presents the best results in whole emergency indications. The long-terms results are multifactorial and depends of additional injuries severity.

Patients with complicated TBD require immediate invasive management to prevent death or injury from rupture or organ malperfusion. The IRAD (International Registry of Acute Aortic Dissections) register confirmed that in 25% of acute B dissection the course is complicated [14]. Trimarchi et al. showed from the same registry that among patients with refractory hypertension (requiring ≥3 different classes of antihypertensive treatment at the maximum tolerated doses), mortality after conservative treatment increased more than 20-fold (35.6% vs. 1.5%; *p*=0.0003) [15]. An alternative, open surgery due to cTBD carries a mortality rate exceeding 30% [16, 17]. The same findings applied to the treatment of RTAA [18, 19]. Advances in technical aspects of TEVAR and enormous experiences gained by dedicated “aortic teams” shifted management from surgical to endovascular repair, contributing to a fourfold increase in early survival in cTBD and RTAA, including also high-risk elderly population [20]. Our results support earlier findings that even in cTBD and RTAA early and medium-term outcomes can be perfect. Although, in our observation, a long-term probability of survival (approximately 60% after 10 years) following cTBD or RTAA is worse than after TAI but still presents a good primary and secondary clinical success rate, much better than treated medically. Previously, in medium-term 5-year observations, it was confirmed that the mortality rate in TEVAR compared to the optimal medical treatment in cTBD was significantly lower (16% vs. 29%; *p*=0.018), even despite the higher risk profile of the TEVAR group [21]. Data from IRAD and INSTEAD-XL (Investigation of Stent grafts in Aortic Dissection with extended length of follow-up) also confirm better 5-year results in patients with cTBD treated with TEVAR [22]. Patel et al. hypothesize that TEVAR may modify the natural course of aortic disease without an unacceptably higher risk of surgery-related death in cTBD [23]. In addition, the recent European guidelines on endovascular treatment of the descending thoracic aorta recommends endovascular repair as the first option in cases of RTAA, provided the anatomical characteristics are suitable (Management of Descending Thoracic Aorta Diseases: Clinical Practice Guidelines of the European Society for Vascular Surgery [CPG-ESVS]); recommendation 23: class I, level of evidence B) [24].

### 4.2. Complications

Endovascular interventions are associated with a risk of serious complications. The most important are endoleaks, stent graft displacement, neurological complications, and retrograde aortic dissection [25–27]. In our group, no patient suffered permanent paraplegia. It is similar to the reported earlier emergency TEVAR cases [2, 20]. A perioperative spinal drainage was not used in our series of emergency interventions. The single case of spinal ischemia (grade 1 according to SVS) and, fortunately, transient paraparesis in our series involved a patient with cTBD who required implantation of 2 grafts. It was proved previously that prosthesis covering the aortic segment longer than 205 mm may increase the risk of spinal ischemia [28, 29]. Stent graft device manipulation within the arch or overstenting of one or more of the great vessels increase the risk of brain injury and ischaemic stroke to 10–15% [30–32]. In our series, two patients (2.6%) developed stroke and in one case it was the cause of death on the 46th day after the procedure.

One of the most serious complications following TEVAR procedures are endoleaks, considered by some authors as a failure of the implantation procedure resulting from incorrect planning. Tokyo Consensus indications emphasizes attention on the length of the LZ, aortic angulation, and calcification [4–6, 33, 34]. In three emergency cases, type I endoleaks directly after the procedures were noted, two of them needed reintervention and another short graft implantation because of significant endoleak and aneurysm extension. In one case we observed hemodynamically nonsignificant type I endoleak. The rare complication are retrograde type A dissection. It may be caused by endovascular prostheses with proximal bare springs, additional balloon dilatation of proximal graft segments, and graft oversizing. We followed strictly expert consensus that oversizing in type B dissection should be avoided [35–38].

The challenging and difficult-to-treat complications are rare erosion of the oesophagus (aorto-oesophageal fistula–AEF) or the left main bronchus [39]. Takeno et al. hypothesize that postoperative aortic disease was the most common cause of AEF, followed by a primary aortic aneurysm, bone ingestion, and thoracic cancer. In our group, one patient presented a primary aorto-oesophageal fistula with a giant aortic aneurysm diameter. The patient after stent graft implantation was operated on due to aorto-oesophageal fistulas with oesophagus plasty but developed sepsis that eventually led to fatal MOF and death on the 19th postoperative day. The second patient developed aorto-oesophageal fistula after previous stent graft implantation for uncomplicated type B dissection in the another center. He underwent complex and multistage treatment including another stent graft implantation, esophageal stenting, and open esophagus repair. Because of the infection's persistence, he was reoperated with graft replacement and aortic arch repair. Unfortunately, the further course was unfavorable and eventually the patient died of sepsis and multiorgan failure.

In 2002, Fillinger et al. proposed the division of the aorta into five landing zones (LZ) to enable proper planning of the TEVAR strategy, including also hybrid treatment [4–6, 33, 34]. Later, authors of the 2004 Tokyo Consensus recommended the minimum length of the aortic pathology-free segment for safe fixation should be >20 mm with LZ aortic diameter >38/40 mm to minimalize the risk of leakage (endoleak I) [4–6, 34, 39–45]. The next expert consensus proposed no stent-graft deployment in patients with a proximal and/or distal landing zone length of less than 25 mm or a maximum diameter of more than 38 mm and no graft oversizing in type B dissection [6]. In rather rare cases if pathology forces to choose LZ 0-1, hemi-arch (LZ 1), or total-arch (LZ 0) debranching precedes safe stent graft implantation. An alternative is a high risk open surgical repair but not in many, even high volume cardiac surgical centers, such emergent operations are routinely performed. Therefore, TEVAR methods seem to be preferable. In our group, in two patients (2.7%) we performed U-shaped carotid-to-carotid prosthesis bypass causes the stent graft distal implantation zone was in LZ 1. Safety criteria of the TEVAR procedure adopted strictly in our center and meeting the recommendations of the Tokyo Consensus including minimal proximal and distal Landing Zone—20 mm (since 2019–25 mm) may have positively impacted results in our center emergent TEVAR.

### 4.3. Limitations

We are aware that the current study has several limitations. First, the retrospective nonrandomized design and analysis of a limited number of patients from a single center reduces the statistical power of the study. The mortality and morbidity rate are very low as well as general outcomes favorable. Therefore, they may not reflect the results of the other centers. Moreover, we must stress that this report was focused predominantly on mortality and morbidity but the quality of life of survivors was not estimated. The latter aspect would increase markedly the significance of this study; therefore, we plan to conduct such a study in the very close future.

## 5. Conclusions

Descending aortic pathologies requiring emergent interventions can be treated by endovascular techniques with optimal results and low morbidity and mortality in an experienced and dedicated team. They are characterized by substantially declined mortality and morbidity, notable including also patients with severe clinical status. Key for primary and secondary clinical success is proper technique planning including minimal distal and proximal Landing Zone strategy.

## Figures and Tables

**Figure 1:** STROBE diagram for various phases of the study (STROBE: strengthening the reporting of observational studies in epidemiology; DAA: descending aorta aneurysm).

**Figure 2:** Probability of survival after TEVAR: (a) total probability and (b) probability in csAAS and TAI subgroups. csAAS: complicated spontaneous acute aortic syndrome; TAI: traumatic aortic injury.

**Table 1:** Demographic data and risk factors.

#	*N* = 74
Age (years)	59.5 (18; 82)
Gender (male/female)	48 (64.8%)/26 (33.2%)
Diabetes mellitus	52 (70.2%)
COPD	27 (36.4%)
Cerebrovascular diseases	12 (16.2%)
History of smoking	57 (77%)
Hypertension	58 (78.3%)
ASA class III to V	60 (81%)
Previous cardiovascular surgery	12 (16.2%)
Critical preoperative state	19 (25.6%)

# continuous variables are expressed as median with range (within bracket) while categorical data as numbers (*n*) with percentage (%). COPD: chronic obstructive pulmonary disease; ASA: American society of anesthesiologists classification.

**Table 2:** Indications and perioperative characteristics.

Indications		Age	Male	LZ^*∗*^	Primary technical success^*∗*^
csAAS *n* = 48	cTBD [*n* = 23]	60.5 (26; 82)	30 (62.5%)	LZ3-4: 21	45/48 (93.7%)
	RTAA [*n* = 23]			LZ2: 26	
	PAU/IH [*n* = 2]			LZ1: 2	

TAI *n* = 23	TAD [*n* = 14], type IV^*∗*^	59 (18; 76)	17 (73.9%)	LZ3-4: 17	23/23 (100%)
	Pseudoaneurysm [*n* = 9], type III			LZ2: 6	

Others *n* = 3	AID [*n* = 1]	50 (35; 66)	1 (33.3%)	LZ3-4: 2	3/3 (100%)
	Fistula [*n* = 2]			LZ2: 1	

Total	*n* = 74	59.5 (18; 82)	48 (64.8%)	LZ3-4: 38	71/74 (95.9%)
				LZ2: 34	
				LZ1: 2	

# continuous variables are expressed as median with range (within bracket) while categorical data as numbers (*n*) with percentage (%); ^*∗*^ according to society of vascular surgery society [4]. csAAS: complicated spontaneous acute aortic syndrome; cTBD: complicated aortic dissection; PAU: penetrating atherosclerotic ulcer; IH: intramural hematoma; RTAA: ruptured descending thoracic aortic aneurysm; TAI: traumatic aortic injury; TAD: traumatic aortic disruption; AID: aortic iatrogenic dissection; LZ: landing zone.

**Table 3:** Primary and secondary clinical success, mortality, and cause of death.

	csAAS	TAI	Others	Total
Primary clinical success^*∗*^	45/48 (93.7%)	23/23 (100%)	2/3 (66.6%)	**70/74 (94.5%)**
Secondary clinical success^*∗*^	44/48 (91.6%)	23/23 (100%)	2/3 (66.6%)	**69/74 (93.2%)**
TEVAR related deaths^*∗*^	0	0	2 (2.6%)	**2 (2.6%)**
<30 days mortality	0	0	1 (1.3%)	**1 (1.3%)**
>30 days mortality	10 (13.5%)	0	1 (1.3%)	**11 (14.8%)**
Causes of death	10 (13.5%)	0	2 (2.6%)	**12 (15.4%)**
*Multiorgan failure*	0	0	2 (2.6%)	**2 (2.6%)**
*Stroke*	1 (1.3%)	0	0	**1 (1.3%)**
*No TEVAR related deaths*	9 (12.1%)	0	0	**9 (12.1%)**

# categorical data are presented as numbers (*n*) with percentage (%); ^*∗*^ according to society of vascular surgery society [4].

**Table 4:** Postoperative complications, other interventions, reinterventions, and causes of death.

Complications	*N* (%)	Mild^*∗*^	Moderate^*∗*^	Severe^*∗*^
Concomitant haemothorax	18 (24.3%)	—	18	—
ARI/hemodialysis	7 (9.4%)	7	—	
Respiratory failure	4 (5.4%)	—	2	2
Mesenteric ischemia	1 (1.3%)	—	—	1
PIS	37 (50%)	37	—	—
Paraplegia	1 (1.3%)	—	1	—
Stroke	2 (2.6%)	—	—	2
Endoleak (type I)	5 (6.8%)			
Early < 24 months	4 (3.9%)	1	2	1
Late > 24 months	1 (1.3%)	—	—	1

Reinterventions	4 (5.2%)			
Early < 24 months	3 (3.9%)			
Late > 24 months	2 (1.3%)			
Paraplegia	1 (1.3%) (spinal cord ischemia grading system—1)^*∗*^			
Stroke	2 (2.6%) (mild and severe)^*∗*^			

ARI: acute renal insufficiency; PIS: postimplantation syndrome. # categorical data are presented as numbers (*n*) with percentage (%); ^*∗*^ according to Society of Vascular Surgery society.

## Data Availability

The data used to support the findings of this study are available from the corresponding author upon request.

## Abbreviations

csAAS: Complicated spontaneous acute aortic syndrome
cTBD: Complicated type B dissection
ID: Iatrogenic dissection
IH: Intramural hematoma
LZ: Landing zone
PAU: Penetrating atherosclerotic ulcer
PIS: Post implantation syndrome
RTAA: Ruptured descending thoracic aortic aneurysm
TAA: Traumatic aortic aneurysm
TAD: Traumatic aortic disruption
TAI: Thoracic aortic injury
TEVAR: Thoracic endovascular aortic repair.

## References

[1] Lee W. A., Matsumura J. S., Mitchell R. S. (2011). Endovascular repair of traumatic thoracic aortic injury: clinical practice guidelines of the Society for Vascular Surgery. *Journal of Vascular Surgery*.

[2] Cambria R. P., Crawford R. S., Cho J. S. (2009). A multicenter clinical trial of endovascular stent graft repair of acute catastrophes of the descending thoracic aorta. *Journal of Vascular Surgery*.

[3] Parker J. D., Golledge J. (2008). Outcome of endovascular treatment of acute type B aortic dissection. *The Annals of Thoracic Surgery*.

[4] Fillinger M. F., Greenberg R. K., McKinsey J. F., Chaikof E. L. (2010). Reporting standards for thoracic endovascular aortic repair (TEVAR). *Journal of Vascular Surgery*.

[5] Mitchell R. S., Ishimaru S., Criado F. J. (2005). Third international summit on thoracic aortic endografting: lessons from long-term results of thoracic stent-graft repairs. *Journal of Endovascular Therapy*.

[6] Czerny M., Schmidli J., Adler S. (2019). Current options and recommendations for the treatment of thoracic aortic pathologies involving the aortic arch: an expert consensus document of the European Association for Cardio-Thoracic surgery (EACTS) and the european society for vascular surgery (ESVS). *European Journal of Cardio-Thoracic Surgery*.

[7] Mitchell M. E., Rushton F. W., Boland A. B., Byrd T. C., Baldwin Z. K. (2011). Emergency procedures on the descending thoracic aorta in the endovascular era. *Journal of Vascular Surgery*.

[8] Harky A., Kai Chan J. S., Ming Wong C. H., Bashir M. (2019). Open versus endovascular repair of descending tho- racic aortic aneurysm disease: a systematic review and meta-analysis. *Annals of Vascular Surgery*.

[9] Richens D., Field M., Neale M., Oakley C. (2002). The mechanism of injury in blunt traumatic rupture of the aorta. *European Journal of Cardio-Thoracic Surgery*.

[10] Buczkowski P., Puslecki M., Stefaniak S. (2017). Post-traumatic acute thoracic aortic injury (TAI)—a single center experience. *Journal of Thoracic Disease*.

[11] Murad M. H., Rizvi A. Z., Malgor R. (2011). Comparative effectiveness of the treatments for thoracic aortic transaction. *Journal of Vascular Surgery*.

[12] Azizzadeh A., Keyhani K., Miller C. C., Coogan S. M., Safi H. J., Estrera A. L. (2009). Blunt traumatic aortic injury: initial experience with endovascular repair. *Journal of Vascular Surgery*.

[13] Böckler D., Riambau V., Coppi G. (2017). Editor’s choice - management of descending thoracic aorta diseases: clinical practice guidelines of the European Society for Vascular Surgery (ESVS). *European Journal of Vascular and Endovascular Surgery*.

[14] Fattori R., Tsai T. T., Myrmel T. (2008). Complicated acute type b dissection: is surgery still the best option?: a report from the international registry of acute aortic dissection. *JACC: Cardiovascular Interventions*.

[15] Trimarchi S., Eagle K. A., Nienaber C. A. (2010). Importance of refractory pain and hypertension in acute type B aortic dissection: insights from the international registry of acute aortic dissection (IRAD). *Circulation*.

[16] Hagan P. G., Nienaber C. A., Isselbacher E. M. (2000). The international registry of acute aortic dissection (IRAD): new insights into an old disease. *JAMA, the Journal of the American Medical Association*.

[17] Suzuki T., Mehta R. H., Ince H. (2003). Clinical profiles and outcomes of acute type B aortic dissection in the current era: lessons from the international registry of aortic dissection (IRAD). *Circulation*.

[18] Girardi L. N., Krieger K. H., Altorki N. K., Mack C. A., Lee L. Y., Isom O. W. (2002). Ruptured descending and thoracoabdominal aortic aneurysms. *The Annals of Thoracic Surgery*.

[19] Barbato J. E., Kim J. Y., Zenati M. (2007). Contemporary results of open repair of ruptured descending thoracic and thoracoabdominal aortic aneurysms. *Journal of Vascular Surgery*.

[20] Jonker F. H., Trimarchi S., Muhs B. E. (2013). The role of age in complicated acute type B aortic dissection. *The Annals of Thoracic Surgery*.

[21] Fattori R., Montgomery D., Lovato L. (2013). Survival after endovascular therapy in patients with type B aortic dissection: a report from the International Registry of Acute Aortic Dissection (IRAD). *JACC: Cardiovascular Interventions*.

[22] Nienaber C. A., Kische S., Rousseau H. (2013). Endovascular repair of type B aortic dissection: long-term results of the randomized investigation of stent grafts in aortic dissection trial. *Circulation: Cardiovascular Interventions*.

[23] Patel A. Y., Eagle K. A., Vaishnava P. (2014). Acute type B aortic dissection: insights from the international registry of acute aortic dissection. *Annals of Cardiothoracic Surgery*.

[24] Goodney P. P., Travis L., Lucas F. L. (2011). Survival after open versus endovascu- lar thoracic aortic aneurysm repair in an observational study of the medicare population. *Circulation*.

[25] Núñez-Gil I. J., Bautista D., Cerrato E. (2015). Registry on aortic iatrogenic dissection (RAID) incidence, management, and immediate- and long-term outcomes after iatrogenic aortic dissection during diagnostic or interventional coronary procedures. *Circulation*.

[26] Von Oppell U. O., Dunne T. T., DeGroot M. K., Zilla P. (1994). Traumatic aortic rupture: twenty-year metaanalysis of mortality and risk of paraplegia. *The Annals of Thoracic Surgery*.

[27] López Espada C., Linares Palomino J. P., Domínguez González J. M. (2021). A multicenter study of emergency endovascular repair of the thoracic aorta: indications and outcomes. *Medicina Intensiva*.

[28] Buczkowski P., Puślecki M., Majewska N. (2019). Endovascular treatment of complex diseases of the thoracic aorta—10 years single centre experience. *Journal of Thoracic Disease*.

[29] Hill A. B., Kalman P. G., Johnston K. W., Vosu H. A. (1994). Reversal of delayed- onset paraplegia after thoracic aortic surgery with cerebrospinal fluid drainage. *Journal of Vascular Surgery*.

[30] Kotelis D., Bischoff M. S., Jobst B. (2012). Morphological risk factors of stroke during thoracic endovascular aortic repair. *Langenbeck’s Archives of Surgery*.

[31] Melissano G., Tshomba Y., Bertoglio L., Rinaldi E., Chiesa R. (2012). Analysis of stroke after TEVAR involving the aortic arch. *European Journal of Vascular and Endovascular Surgery*.

[32] Patel H. J., Shillingford M. S., Williams D. M. (2007). Survival benefit of endovascular descending thoracic aortic repair for the high-risk patient. *The Annals of Thoracic Surgery*.

[33] Criado F. J., Clark N. S., Barnatan M. F. (2002). Stent graft repair in the aortic arch and descending thoracic aorta: a 4-year experience. *Journal of Vascular Surgery*.

[34] Criado F. J., Abul-Khoudoud O. R., Domer G. S. (2005). Endovascular repair of the thoracic aorta: lessons learned. *The Annals of Thoracic Surgery*.

[35] Zarins C. K., White R. A., Schwarten D. (1999). AneuRx stent graft versus open surgical repair of abdominal aortic aneurysms: multicenter prospective clinical trial. *Journal of Vascular Surgery*.

[36] Gottardi R., Funovics M., Eggers N. (2008). Supra-aortic transposition for combined vascular and endovascular repair of aortic arch pathology. *The Annals of Thoracic Surgery*.

[37] Ma T., Dong Z. H., Wang S., Meng Z. Y., Chen Y. Y., Fu W. G. (2018). Computational investigation of interaction between stent graft and aorta in retrograde type A dissection after thoracic endovascular aortic repair for type B aortic dissection. *Journal of Vascular Surgery*.

[38] Mosquera V. X., Marini M., Fraga-Manteiga D., Gulias D., Cuenca J. J. (2016). Repair of late retrograde type a aortic dissection after tevar: causes and management. *Journal of Cardiac Surgery*.

[39] Takeno S., Ishii H., Nanashima A., Nakamura K. (2020). Aortoesophageal fistula: review of trends in the last decade. *Surgery Today*.

[40] Moore R. D., Brandschwei F. (2001). Subclavian-to-carotid transposition and supracarotid endovascular stent graft placement for traumatic aortic disruption. *Annals of Vascular Surgery*.

[41] Peterson B. G., Eskandari M. K., Gleason T. G., Morasch M. D. (2006). Utility of left subclavian artery revascularization in association with endoluminal repair of acute and chronic thoracic aortic pathology. *Journal of Vascular Surgery*.

[42] Riesenman P. J., Farber M. A., Mendes R. R., Marston W. A., Fulton J. J., Keagy B. A. (2007). Coverage of the left subclavian artery during thoracic endovascular aortic repair. *Journal of Vascular Surgery*.

[43] Belczak S. Q., Silva E. S., Klajner R., Puech-Leao P., De Luccia N. (2017). Type ii endoleaks, left-arm complications, and need of revascularization after left subclavian artery coverage for thoracic aortic aneurysms endovascular repair: A systematic review. *Annals of Vascular Surgery*.

[44] Hajibandeh S., Hajibandeh S., Antoniou S. A., Torella F., Antoniou GA. (2016). Meta-analysis of left subclavian artery coverage with and without revascularization in thoracic endovascular aortic repair. *Journal of Endovascular Therapy*.

[45] Vriend J. W., Mulder B. J. (2005). Late complications in patients after repair of aortic coarctation: implications for management. *International Journal of Cardiology*.

